This article has been retracted.

# Applying Blockchain Technology in Network Public Opinion Risk Management System in Big Data Environment

**DOI:** 10.1155/2023/5212712

**Published:** 2023-03-10

**Authors:** Zhenqing Luo, Cheng Zhang

**Affiliations:** ^1^School of Journalism and Communication, Renmin University of China, Beijing 100872, China; ^2^College of Movie and Media, Sichuan Normal University, Chengdu 610066, China

## Abstract

Network public opinion represents public social opinion to a certain extent and has an important impact on formulating national policies and judgment. Therefore, China and other countries attach great importance to the study of online public opinion. However, the current researches lack the combination of theory and practical cases and lack the intersection of social and natural sciences. This work aims to overcome the technical defects of traditional management systems, break through the difficulties and pain points of existing network public opinion risk management, and improve the efficiency of network public opinion risk management. Firstly, a network public opinion isolation strategy based on the infectious disease propagation model is proposed, and the optimal control theory is used to realize a functional control model to maximize social utility. Secondly, blockchain technology is used to build a network public opinion risk management system. The system is used to conduct a detailed study on identifying and perceiving online public opinion risk. Finally, a Chinese word segmentation scheme based on Long Short-Term Memory (LSTM) network model and a text emotion recognition scheme based on a convolutional neural network are proposed. Both schemes are validated on a typical corpus. The results show that when the system has a control strategy, the number of susceptible drops significantly. Two days after the public opinion is generated, the number of susceptible people decreased from 1,000 to 250; 3 days after the public opinion is generated, the number of susceptible people stabilized. 2 days after the public opinion is generated, the number of lurkers increased from 100 to 620; 3 days after the public opinion is generated, the number of lurkers stabilized. The data demonstrate that the designed isolation control strategy is effective. Changes in public opinion among infected people show that quarantine control strategies played a significant role in the early days of Corona Virus Disease 2019. The rate of change in the number of infections is more affected when quarantine controls are increased, especially in the days leading up to the outbreak. When the system adopts the optimal control strategy, the influence scope of public opinion becomes smaller, and the control becomes easier. When the dimension of the word vector of emergent events is 200, its accuracy may be higher. This method provides certain ideas for blockchain and deep learning technology in network public opinion control.

## 1. Introduction

Since the 21st century, information technology has been effectively used in all aspects of social life, and significant changes have taken place in the amount and state of information. Increasing information appears in this era, and information explosion has become a distinctive feature. Applying information technology in society has generated massive data and information resources. The collection, dissemination, storage, and processing of resources have become a common concern of communities and enterprises. Internet of things, big data, and blockchain technologies are increasingly used to mine and analyze a wealth of data. Therefore, new technologies affect people's work and lifestyle, bringing new methods and challenges to monitoring and processing network public opinion. As we all know, the Internet changes people's lives and makes life more efficient and faster. Social networks have become a critical platform for network users to express their opinions and vent their emotions [1, 2]. Social networks show the characteristics of fast communication speed and wide communication range and have an even more significant impact on ordinary people and society. People discuss and communicate social events through forums, microblogs, WeChat, and other instant-messaging tools. Compared with traditional public opinion, social network public opinion formed in this way realizes free expression and communication and reveals people's true feelings. Because social networks can easily promote the interaction between Internet users, this interaction makes the emergence and evolution of public opinion more rapid and the dissemination of public opinion more random and complex. However, meanwhile, the rapid development of social networks has accelerated the spread of opposing public views, such as false information and network rumors. Under certain circumstances, it will bring many unstable factors to society and weaken the government's credibility, thus affecting the government's decision-making and reducing the social identity of society's mainstream values. Therefore, the research on social network public opinion communication has become a widespread concern in the academic community [3]. As a product of the rapid development of the Internet and network technology in the era of big data, online public opinion is a more real “public voice” that the government cannot ignore. It enriches the way people express their attitudes and changes the way people live and work. The government can more accurately obtain the needs of the public and understand the focus of the public by analyzing public opinion on the Internet. Additionally, in order to maintain social stability and enhance the image of the government, relevant departments also need to intervene and control online public opinion. Therefore, studying the factors affecting the laws of network public opinion plays an important role in understanding the dissemination mechanism of network public opinion, intervening in public opinion, reducing or restricting the development of negative network public opinion, and maintaining social stability.

Researchers in the field of network public opinion control have also done a lot of work. Li et al. [4] studied the evolution of communities in the process of public opinion dissemination and proposed a public opinion evolution model for online communities. The highlight of this model is that, on the one hand, it realizes the research on the evolution of public opinion in the dynamic network; on the other hand, unlike other public opinion evolution models, this model focuses on the law of increase and decrease of the number of communities in the process of public opinion evolution. Fu et al. [5] pointed out that the occurrence of hot social events caused fluctuations and changes in public sentiment. The rapid development of online social platforms and networks has made individual interactions more intense, escalating public sentiment into public opinion. However, the exploration of online public opinion lacks consideration of individual emotions. Firstly, quantitative representations of attitudes and emotions are elaborated. The formation and dissemination process of online public opinion is analyzed based on factors such as the individual's willingness to express, the individual's ability to express, the perceived value of attitude, and the probability of attitude change. A dissemination model of online public opinion considering individual emotional factors is constructed. Zhang et al. [6] pointed out that with the rapid development of the Internet, social media networks have become the main platform for people to express their opinions. In addition, online public opinion has a considerable impact on society. Therefore, the dissemination process of network public opinion is studied and analyzed. A model of media and interpersonal relationships is proposed. The model considers the influence of media communication and interpersonal relationships on opinion diffusion. He et al. [7] pointed out that natural disasters have long plagued people's normal life. How to effectively identify and evaluate areas affected by natural disasters and further control network public opinion is of great significance. In 2017, the flood disaster in Hunan Province was taken as an example. Based on the data source of Weibo, combined with text analysis and image analysis techniques, the scope of natural disasters was determined. Then, sentiment and correlation analysis methods are used to study the network public opinion in the disaster area. Cao et al. [8] pointed out that the spread of public opinion in the rough network of third-party payments may endanger the economic stability of the platform. Therefore, assessing the risk of online public opinion dissemination is imminent. The research on the characteristics of the third-party payment rough network public opinion dissemination is used to determine the essence of the risk assessment of network public opinion dissemination; that is, the evaluation of important nodes in the network and the risk of customer mining. A game theory-based node selection model and a node search algorithm are established. In order to overcome the threat posed by online public opinion, the state, enterprises, and society must actively protect cyberspace. Related research on Internet public opinion is investigated. The research on network security management and public opinion diffusion has achieved rich results in both theory and application. These results provide a solid foundation for this work. However, these results still lack a systematic and complete analysis of public security incidents to a certain extent. The research results of public opinion management are limited to simple conceptual interpretation and application. There is no in-depth analysis of the public opinion management and impact of emergencies, and there is no research on the monitoring, early warning, and prevention of security crisis events at the system level.

Therefore, the present work constructs a control model with social utility maximization objective function by using the method of optimal control theory and proves the accuracy of the solution and the effectiveness of the strategy through simulation. In addition, a network public opinion risk management system is proposed based on network public opinion risk management, elastic management, and blockchain technology, followed by a detailed analysis on the intelligent classification ledger of network public opinion risk identification and perception, risk association tree, and smart contract. The research reported here innovatively studies the spread of public opinion from the dynamic theory of differential equations. It constructs an objective function control model with social utility maximization from cybernetics.

## 2. Construction and Design of the Optimal Isolation Strategy of Network Public Opinion in an Enclosed Environment

### 2.1. Analysis of Network Public Opinion and Infectious Disease Transmission Model

“Public opinion” and “network public opinion” are two concepts with Chinese characteristics. Their ideas and related systems have a long history in China. In the books of the last century, “public opinion” is interpreted as “the will of the people”. Public opinion research is an interdisciplinary research field combining natural science and social science. Basic theoretical research on public opinion began in the 21st century [9, 10]. Generally speaking, scholars' understanding of public opinion is divided into two aspects: narrow sense and broad sense. In the narrow sense, public opinions refer to the social and political attitudes of the people towards the national management and decision-makers in the context of a particular social space. In a broad sense, public opinions refer to people's living background and environment, overall living, and personal subjective will. With the rapid popularization of Internet technology globally, the network is gradually recognized as the “fourth media” after newspapers, radio, and television. The network has become one of the leading media carrying public social opinion, and network public opinion, as a new concept, is put forward under this social background [11]. Compared with traditional public opinion, network public opinion has three characteristics: 1. network public opinion comes from a wide range of sources; 2. network public opinion is obtained directly; 3. network public opinion communication has concealment and deviation; 4. the formation of network public opinion is sudden [12, 13].  Figure 1 shows the characteristics and evolution mechanism of network public opinion.

The characteristics of network public opinion can be divided into four points: 1. anonymity and diversification. In the Internet, people cannot use their real identity but use a virtual identity to appear in the network. This virtual identity provides a space for the public to publish their own topics and opinions and promotes the diversification of public opinion. 2. Immediacy and interactivity. The network can publish some of the latest major social events in a very short period. Netizens can learn about current events and express their views on events in the fastest time and leave their own comments on the corresponding online platforms. Its timeliness is a function that traditional paper media does not have. The real-time nature of the network makes the dissemination of network public opinion faster, and public social opinion can be quickly collected, and corresponding measures can be taken. 3. Difficulty controllability and controllability. The emergence of the Internet makes the dissemination of information no longer limited by time and space. Although this kind of unrestricted brings certain convenience, it also greatly challenges the relevant departments to control network public opinion. 4. Extensiveness and limitations. The rapid spread of online public opinion, the wide range of influence, and the large coverage area are beyond the reach of traditional media. Therefore, it largely replaces many functions of traditional media. However, there are still some people in society who are not regular netizens. These groups are not greatly affected by the network. Therefore, online public opinion has certain limitations on the audience. The network public opinion evolution mechanism of social emergencies can be divided into three stages. 1. Public discussion stage. From the generation of netizens' opinions to the formation of the network public opinion field, the outbreak of network public opinion is determined by the coupling effect of touch point events and the environment. As a window of social contradictions and a release state of public emotional backlog, social emergencies have the characteristics of suddenness, destruction, and irritation. Driven by multiple potential logics such as politics, economy, culture, social life, and media, and influenced by individual factors such as perception judgment and mental schema, individuals in public will generate corresponding emotions, attitudes, and opinions when triggered. The Internet is used to express emotions or demands. 2. Public controversy stage. The development and transfer of public opinion on the Internet is analyzed based on Kurt Koffka's psychophysical field theory. As a new public domain, the materiality of the Internet provides a physical field for public opinion to brew and develop. It also provides a psychological field for the climate of public opinion due to the intersection of political ideology, social values, media culture, and other factors. Therefore, the network public opinion field is complex and changeable, with many symbiotic effects. When group opinions on social emergencies are gathered and a clear mainstream of public opinion is formed, the group norms and group pressures of online public opinion groups are revealed under the influence of the media “habituation” and the social field of network communication. At this time, public behavior and emotions in public opinion turmoil are not only caused by individual characteristics but also affected by the situation of network public opinion groups. 3. The organizational decision-making stage is when network public opinion fades and transitions to social behavior. Since it has entered the stage of dialogue with the official, the mainstream media at this time can obtain core information sources, verify facts, and clarify rumors. Under the joint guidance of the official and mainstream media, online public opinion is fading.

Based on the similarity between the spread of public opinion information and the spread mechanism of infectious diseases, the infectious disease model is expanded to the spread field of network public opinion. The Susceptible Infected Recovered (SIR) model proposed by other researchers is a representative dynamic model of infectious diseases. The SIR model divides the research objects into three categories according to the spread characteristics of infectious diseases and environmental conditions: the susceptible person, the infected person, and the removed person. Among them, the susceptible person represents the individuals who are not infected by the disease but may be infected in the future. The infected person represents the infected and infectious individuals. The removed person represents the individuals immune to such conditions [14, 15]. The ordinary differential equation of the SIR model can be written as

(1) $$\begin{array}{c} \left\{\begin{array}{c} \dot{S}=-\beta SI,\\ \dot{I}=\beta SI-\gamma I,\\ \dot{R}=\gamma I. \end{array}\right. \end{array}$$

In (1), $\dot{S}$ denotes the susceptible person, $\dot{I}$ refers to the infected person, and $\dot{R}$ denotes the removed person. Besides, *β* stands for the proportional coefficient between the number of susceptible persons infected by each infected person and the number of susceptible persons per unit time, and *γ* signifies the ratio between the number of rehabilitated persons and infected persons per unit time. The threshold *R*_0_ is an essential variable in the infectious disease model, and *R*_*0*_ = 1 is the basis for judging whether public opinion communication will die. When *R*_*0*_ < 1, communication will gradually disappear; in other words, with the progress of communication and the passage of time, all individuals who know public opinion will eventually be removed from the system. When *R*_*0*_ > 1, public opinion will spread within a specific range and will not disappear.

The core of modern control theory is the optimal control theory. The problem of the optimal control system can be summarized as focusing on the dynamic design and motion process in the steady state and finding the optimal scheme from many feasible control schemes. When the motion state of the system changes, that is, from an initial state to a target state, the performance index of the system is the best [16, 17]. Equation (2) indicates the mathematical expression of the optimal control problem.

(2) $$\begin{array}{c} \min J\left(u\left(.\right)\right)=\int_{0}^{T}F\left(x\left(t\right),u\left(t\right),t\right)\text{d}t. \end{array}$$

In (2), *u*(*t*) is the optimal control vector; *J*(*u*(.)) is the performance index; *x*(*t*) is the final state.

The corresponding equation of state containing order *n* can be written as

(3) $$\begin{array}{c} x=f\left(x,u,t\right). \end{array}$$

The initial conditions can be expressed as

(4) $$\begin{array}{c} x\left(t_{0}\right)=x_{0}. \end{array}$$

In equation (4), *x*(*t*) ∈ *R*^*n*^, *t* ∈ [*t*_0_, *T*], and *u*(*t*) ∈ Ω⊆*R*^*m*^. The vector function *f*(*x*, *u*, *t*) is a continuous function of *x*(*t*), *u*(*t*), and *t*, which is continuously differentiable.

### 2.2. Design of the Network Public Opinion Communication Impact Model with an Isolation Control Strategy

The research environment adopted here is a relatively closed environment, in which the number of people almost remains unchanged, and no people are moving in and out. This public opinion environment is described through the basic infectious disease SIR model. The most significant difference between the spread of information and infectious diseases lies in the different removal mechanisms. The spread of data is a manifestation of the disseminator's subjective initiative. When an uninformed person receives a message, they will think about whether they want to spread the message. This thinking process has a great relationship with the uninformed person's educational background, judgment ability, and personal interest. When an unknown person receives a message, they will hold a confident hesitant attitude, which interferes with message transmission. Considering this delay, the new variable lurker *L* is introduced into the original infectious disease SIR model to construct a control model. In addition, the isolation strategy is utilized to control the development of public opinion after the outbreak of public opinion to minimize the number of network public opinion communicators until they disappear on the premise of minimum cost [18].

Yang and Yu [19] set up a model, in which the objects were divided into four groups, which were respectively disjointed groups (vulnerable individuals who are not aware of a specific network public opinion), the imperceptibly infected group (individuals are thinking about network public opinion, but do not take any action), the group of infected objects (those who spread public opinions through social interaction), and the recovery group (those who know the public opinion but choose not to spread it to others). This model is also used for reference in this study. The basic assumptions of the model are as follows. 1. The main manifestations of the modes of network public opinions contain comments, blogs, microblogs, aggregate news, news posts, and reprints. 2. According to the SIR model's population classification and transmission law, it is assumed that the use of isolation strategy in the public opinion environment can reduce the density of infected people. To facilitate the derivation of the model, it is also assumed that there is a natural immunization rate in the model. Based on the above assumptions, individuals are categorized into different types according to their understanding and communication status of public opinion information. The contact between different kinds of individuals can promote the transmission, diffusion, or extinction of messages, thus changing the attributes of individuals to varying degrees. Let *S*=*S*(*t*)/*N* ≥ 0, *L*=*L*(*t*)/*N* ≥ 0, *I*=*I*(*t*)/*N* ≥ 0, and *R*=*R*(*t*)/*N* ≥ 0, and this situation can be presented as Figure 2.

Network public opinion will get widespread attention and spread rapidly, reaching a climax stage at an almost straight-up speed, that is, the public opinion outbreak stage. It has no transition period between the occurrence and outbreak of public opinion. After the outbreak of online public opinion, due to the follow-up of traditional media and official intervention, the speed of follow-up will have a transition period of public opinion development. During this transition period, if the follow-up speed is fast enough, the network public opinion will quickly enter the recession stage. If the follow-up speed is slow, the network of public opinion will go through a long transition stage; that is, the number of people interested in public opinion will remain relatively large for a long time. If the outside information is improperly involved, or there is a special group to excite the incident. The dissemination of network public opinion will also go through a stage of spreading growth. At this stage, the number of followers of the public opinion continues to increase or maintains a relatively large number in a longer event and enters a recession period with the occurrence of other hot issues.

Based on the above analysis, the public opinion communication model, including the incubation period can be expressed as

(5) $$\begin{array}{c} \text{s}.\text{t}.\left\{\begin{array}{c} \dot{S}=-\beta SI-u_{S}S,\\ \dot{L}=\beta SI-u_{L}L,\\ \dot{I}=u_{L}L-u_{I}I,\\ \dot{R}=u_{s}S+u_{I}I,\\ S\left(0\right)\geq 0,L\left(0\right)\geq 0,I\left(0\right)\geq 0,R\left(0\right)\geq 0. \end{array}\right. \end{array}$$

In (5), *β* stands for the infection rate, meaning the probability that the susceptible person *S* contacts the infected person *I* at *t* time to know the public opinion information, and *βSI* represents that a part of the susceptible people *L* contacts the public opinion information of the infected person *I* at *t* time. Besides, *u*_*L*_ refers to the conversion rate, indicating the conversion coefficient from a lurker to an infected at *t* time, and *u*_*L*_*L* denotes the population in which some lurkers enter the population of the infected *I* at *t* time. Moreover, *u*_*I*_ represents the removal rate, referring to the coefficient corresponding to the *t* time when the infected person *I* enters the immune population, and *u*_*S*_ indicates the natural immune rate. For example, scholars with attainments in a certain field can identify the authenticity of public opinion information, and such people do not easily spread information [20, 21].

When public opinion breaks out, how to control public opinion quickly and effectively becomes the focus of attention. The postulated condition of this paper is to manipulate public opinion in a relatively closed network environment. The isolation strategy is adopted to install gatekeepers in the network, thus strengthening the daily monitoring of network communication content. Any problems will be masked and deleted [22, 23]. Here, the variable *u* is introduced into the model to describe the isolation of public opinion. Correspondingly, the control system can be written as

(6) $$\begin{array}{c} \text{s}.\text{t}.\left\{\begin{array}{c} \dot{S}=-\beta SI-u_{S}S,\\ \dot{L}=\beta SI-u_{L}L,\\ \dot{I}=u_{L}L-\left(u_{l}+u\right)I,\\ R=u_{s}S+u_{l}I,\\ S\left(0\right)\geq 0,L\left(0\right)\geq 0,I\left(0\right)\geq 0,R\left(0\right)\geq 0,\\ 0\leq u\leq u_{\max}\leq 1. \end{array}\right. \end{array}$$

In (6), *u* represents the isolation rate, and *u* ∈ (0, *u*_max_); *u*=0 represents that the isolation strategy is not adopted; *u*=*u*_max_ indicates that the isolation strategy is maximized, where 0 ≤ *u* ≤ *u*_max_ ≤ 1.

Any communication has a communication balance point *R*_0_, which directly plays a decisive role in the communication situation of the system. Here, the system's threshold is calculated by (6). Equation (6) satisfies the relationship shown in (7)-(11). Only the system composed of the first three equations in (6) is considered to simplify the model.

(7) $$\begin{array}{c} S=\frac{S\left(t\right)}{N}\geq 0, \end{array}$$

(8) $$\begin{array}{c} L=\frac{L\left(t\right)}{N}\geq 0, \end{array}$$

(9) $$\begin{array}{c} I=\frac{I\left(t\right)}{N}\geq 0, \end{array}$$

(10) $$\begin{array}{c} R=\frac{R\left(t\right)}{N}\geq 0, \end{array}$$

(11) $$\begin{array}{c} R=1-S-L-I. \end{array}$$

If *x*=(*L*, *I*, *S*)^*T*^, the control system can be reorganized into the form shown in

(12) $$\begin{array}{c} \frac{\text{d}x}{\text{d}t}=\tilde{F}\left(x\right)\tilde{V}\left(x\right). \end{array}$$

In (12), $\tilde{F}\left(x\right)$ represents the outflow rate of a new infection, and $\tilde{V}\left(x\right)$ refers to the conversion rate of individual outflow or entry into each category. $\tilde{F}\left(x\right)$ can be written in the form represented by (13), and $\tilde{V}\left(x\right)$ can be presented as the form shown by (14).

(13) $$\begin{array}{c} \tilde{F}\left(x\right)=\left(\begin{array}{c} \beta SI\\ 0\\ 0 \end{array}\right), \end{array}$$

(14) $$\begin{array}{c} \tilde{V}\left(x\right)=\left(\begin{array}{c} u_{L}L\\ -u_{L}L+\left(u_{I}+u\right)I\\ \beta SI+u_{S}S \end{array}\right). \end{array}$$

The threshold *R*_*0*_, that is, the regeneration matrix, is defined as *FV*^−1^, where *F* and *V* are the Jacobian matrices, which can be written as (15) and (16).

(15) $$\begin{array}{c} V=\left(\frac{\partial {\bar{V}}_{1}}{\partial X_{1}}\left(X_{0}\right)\right),\;1\leq i,j\leq 2, \end{array}$$

(16) $$\begin{array}{c} F=\left(\frac{\partial {\bar{F}}_{1}}{\partial X_{1}}\left(X_{0}\right)\right),\;1\leq i,j\leq 2, \end{array}$$

*X*_0_ is the disease-free equilibrium of (16), and it satisfies

(17) $$\begin{array}{c} X_{0}={\left(\begin{array}{ccc} 0 & 0 & 1 \end{array}\right)}^{T}. \end{array}$$

Then, there are

(18) $$\begin{array}{c} F=\left(\begin{array}{cc} 0 & \beta \\ 0 & 0 \end{array}\right),\\ V=\left(\begin{array}{cc} u_{L} & 0\\ -u_{L} & u_{1}+u \end{array}\right),\\ FV^{-1}=\left(\begin{array}{cc} \frac{\beta }{\left(u_{I}+u\right)} & \frac{\beta }{\left(u_{I}+u\right)}\\ 0 & 0 \end{array}\right). \end{array}$$

According to the spectral radius *ρ*(*FV*^−1^)=max_1≤*i*≤2_|*λ*_*i*_| (|*λ*_*i*_| represents the maximum eigenvalue of the regeneration matrix), the threshold can be calculated, as shown in

(19) $$\begin{array}{c} R_{0}=\frac{\beta }{\left(u_{1}+u\right)}. \end{array}$$

According to the threshold value obtained by (19), the isolation control strategy used in the control system can effectively reduce the threshold value. When the threshold value is less than 1, public opinion will continue to spread over time, all individuals who know public opinion information in the system will be removed from the system, and the spread of public opinion will be effectively controlled.

Based on the above analysis, after the outbreak of public opinion, it is necessary to further analyze the optimal control strategy of the model. This paper considers the maximization of the social utility of public opinion information dissemination control from the following two aspects. The first aspect is to minimize the number of infected individuals; the second aspect is to minimize the cost of the control process. Here, the performance index is used to judge the system's performance, as shown in

(20) $$\begin{array}{c} J\left(u\right)\int_{0}^{1}\left[I+\frac{\alpha u^{2}}{2}\right]\text{d}t. \end{array}$$

In (20), *αu*^2^/2 denotes the cost of adopting a quarantine policy, and *α* refers to the cost weight coefficient in the control process.

Therefore, the research goal is transformed into finding the optimal purpose so that the relationship shown in (21) holds.

(21) $$\begin{array}{c} J\left(u^{*}\right)=\min_{\Omega }J\left(u\right). \end{array}$$

In (21), *u* is a function related to *t* (*t* ∈ (0, *t*_*f*_)), and the set of control constraints is denoted as Ω={*u*/0 ≤ *u* ≤ *u*_max_ ≤ 1}.

The optimal control problem can be described as

(22) $$\begin{array}{c} \min J=\int_{0}^{t}\left[I+\frac{1}{2}\alpha u^{2}\right]\text{d}t,\\ \text{s}.\text{t}.\left\{\begin{array}{c} S=-\beta SI-u_{S}S,\\ L=\beta SI-u_{L}L,\\ I=u_{L}L-\left(u_{l}+u\right)I,\\ S\left(0\right)\geq 0,L\left(0\right)\geq 0,I\left(0\right)\geq 0,\\ 0\leq u\leq u_{\max}\leq 1. \end{array}\right.. \end{array}$$

Here, the optimal control system is constructed by taking the differential equation system as the constraint condition of the objective function, and it is not difficult to see that the optimal control system has an optimal solution. Pontryagin's maximum principle [24, 25] provides the necessary conditions for optimal control. At this time, the optimal control problem can be transformed into the minimum Hamiltonian function problem [26–29]. The corresponding cross-sectional conditions will change when the state equation changes or the terminal conditions change. At this time, the maximum principle is used to explore the optimal value problem.

Equation (23) indicates the Hamiltonian function.

(23) $$\begin{array}{c} H=I+\frac{1}{2}\alpha u^{2}+\lambda_{s}\left(-\beta SI-u_{s}S\right)+\lambda_{L}\left(\beta SI-u_{L}L\right)+\lambda_{I}\left(u_{L}L-\left(u_{I}+u\right)I\right). \end{array}$$

In (23), *λ*_*s*_, *λ*_*L*_, and *λ*_*l*_ are instrument variables.

According to the maximum theorem, *λ*_*s*_, *λ*_*L*_, and *λ*_*l*_ satisfy

(24) $$\begin{array}{c} \lambda_{s}=-\frac{\partial H}{\partial S},\lambda_{L}=-\frac{\partial H}{\partial L},\lambda_{l}=-\frac{\partial H}{\partial I}, \end{array}$$

(25) $$\begin{array}{c} \lambda_{S}\left(t_{f}\right)=\lambda_{L}\left(t_{f}\right)=\lambda_{l}\left(t_{f}\right)=0. \end{array}$$

Substitute *H* into (24), and the costate equation and transect conditions are as (29) ∼ (30).

(26) $$\begin{array}{c} \lambda_{s}=\beta I\left(\lambda_{s}-\lambda_{I}\right)+u_{s}\lambda_{s}, \end{array}$$

(27) $$\begin{array}{c} \lambda_{L}=u_{L}\left(\lambda_{L}-\lambda_{l}\right), \end{array}$$

(28) $$\begin{array}{c} \lambda_{l}=-1+\beta S\left(\lambda_{s}-\lambda_{L}\right)+\left(u_{l}+u\right)\lambda_{l}, \end{array}$$

(29) $$\begin{array}{c} \lambda_{S}\left(t_{f}\right)=\lambda_{L}\left(t_{f}\right)=\lambda_{l}\left(t_{f}\right)=0. \end{array}$$

The optimal control law can be described as

(30) $$\begin{array}{c} u^{*}=\left\{\begin{array}{cc} 0, & \text{if}\frac{\lambda_{I}I}{\alpha }<0,\\ \frac{\lambda_{I}I}{\alpha }, & \text{if 0}\leq \frac{\lambda_{I}I}{\alpha }<u_{\max|},\Rightarrow u=\min\left\{u_{\max},\max\left\{\begin{array}{cc} 0, & \frac{\lambda_{I}I}{\alpha } \end{array}\right\}\right\},\\ u_{\max}, & \text{if}\frac{\lambda_{l}I}{\alpha }u_{\max}. \end{array}\right. \end{array}$$

In (30), *I*,*λ*_*I*_ is an auxiliary variable.

### 2.3. Design of the Network Public Opinion Risk Management System Based on Blockchain

The control objective of the public opinion risk management information system is to find potential public opinion risks, bear public opinion appropriately, and control public opinion within an acceptable range [30–32]. The subject of public opinion control can choose appropriate public opinion risk response strategies and formulate and implement action plans.  Figure 3 shows the framework of the network public opinion risk management system.

The study of relevant literature found that the current standard risk management systems have the following two defects. The first is that the data security is low, and the second is that the data security is difficult to guarantee [33]. Based on the above analysis, a network public opinion risk management system is proposed, including the public opinion risk management system and blockchain data assurance system. The public opinion risk management system architecture designed here is divided into four modules, i.e., public opinion risk perception and identification, public opinion risk analysis, public opinion risk response, and public opinion risk report.  Figure 4 illustrates the network public opinion early warning system.

The association tree is used to dynamically track the public opinion risk according to the risk level, establish the public opinion risk intelligent ledger, and design the public opinion risk performance management table. In the public opinion risk smart contract, the public opinion registration form is formed in the process of public opinion risk identification, and the contract is updated in the process of public opinion risk and public opinion analysis. Public opinion risk smart contracts are divided into three categories: public opinion risk summary project ledger, public opinion risk analysis ledger, and public opinion risk response ledger. The blockchain-based public opinion risk smart ledger has nine key attributes: (1) public opinion event ID; (2) description of public opinion; (3) classification of public opinion; (4) trigger threshold; (5) public opinion status; (6) risk level; (7) probability of public opinion outbreak; (8) public opinion influence; (9) public opinion response plan.

Figure 5 reveals the public opinion risk association tree constructed here.

In Figure 5, the transaction tree maintains transactions in specific blocks. The receipt tree is used to save the detailed data of multiple transactions. The public opinion risk association tree is used to keep the relationships in the ledger. Block 16,3845 is written into the public opinion risk analysis ledger and public opinion risk response ledger. Public opinion risk events, public opinion risk analysis, and public opinion risk response are responded based on the risk hash value.

### 2.4. Simulation Condition Setting

The numerical simulation method analyzes and discusses the model based on theoretical research. During the verification, the parameters are set as *β*=0.04, *u*_*s*_=0.005, *u*_*L*_=0.05, and *u*_*I*_=0.002. To simulate the control results, the public opinion control cycle is set as nine days; under the initial conditions, *S*(0)=1000, *L*(0)=90, and *I*(0)=5.

## 3. Algorithm Test and Simulation

### 3.1. Simulation Results of the Social Network Public Opinion Communication System Based on Empirical Analysis

Figure 6 illustrates the operation results of the public opinion diffusion degree of the social network.

As shown in Figure 6(a), with the improvement of online cultural publicity, the diffusion of public opinion on social networks has changed to a certain extent. This demonstrates that online artistic advertisement has a particular impact on controlling the spread of public opinion events, but the strength is limited. According to Figure 6(b), when the popularity and credibility of opinion leaders increase, the influence of opinion leaders on Internet users can hinder and delay the spread and diffusion of public opinion on social networks. Therefore, it is negatively correlated with the distribution of public opinion on social networks. It proves that the guidance of opinion leaders to netizens is also gradually weakening. Compared with the influence of online cultural publicity, the popularity and credibility of opinion leaders have a more significant impact on the diffusion of social network public opinion. In Figure 6(c), in the beginning, the public opinion diffusion of social networks with high sensitivity to public opinion events increases more. It takes less time than those with low sensitivity. With time, the decline rate is also significant. The reason is that after the outbreak of public opinion events with high sensitivity, the government intervention is more robust and faster, and the spread of public opinion on social networks will be restrained in a short time.

### 3.2. Algorithm Test

Figure 7 shows the track of the network public opinion communication system under the condition of no control.

In Figure 7, in the initial stage of public opinion appearance, when there is no interference control, the number of susceptible persons decreases significantly. Two days after the public opinion is generated, the number of susceptible people is reduced from 1,000 to 300. After three days of public opinion, the number of susceptible persons stabilized. Two days after the public opinion is generated, the number of lurkers increased from 100 to 820. After three days of public opinion, the number of lurkers stabilized. This trend is consistent with reality. Many public opinions spread on the Internet satisfy the curiosity of the unknown and provide information for further disseminating public opinion information.

Figure 8 shows the trajectory of network public opinion dissemination in the system with isolation strategy when the cost weight coefficient in the objective function *α* is two and the upper control limit (UCL) *u*_max_ = 0.1.  Figure 9 displays the trajectory of network public opinion communication in the system with isolation strategy when the cost weight coefficient *α* in the objective function equals two and UCL *u*_max_ = 0.3.

In Figure 8, when the system has a control strategy, the number of susceptible people drops significantly. Two days after the public opinion is generated, the number of susceptible people is reduced from 1,000 to 250. After three days of public opinion, the number of susceptible persons stabilized. Two days after the public opinion is generated, the number of lurkers increases from 100 to 620. After three days of public opinion, the number of lurkers stabilized. When there is a control strategy, the growth rate of public opinion-infected people is slower than when there is no control. The data demonstrate that the isolation control strategy is effective. When the optimal control parameters are used in the control plane, the number of people infected with public opinion is significantly reduced, the peak value is also significantly reduced, and the duration of public opinion is significantly shorter. The data shows that the influence of online public opinion has become smaller, and its control has become easier. In the early days of the Corona Virus Disease 2019 outbreak, the strategy of quarantine control is evident. After adding quarantine controls, the rate of change in the number of infected people is significantly affected. Implementing control in the early stage of the outbreak of public opinion can quickly achieve better results, restrain the wanton spread of public opinion, and reduce unnecessary losses. The data show that the higher the upper limit of isolation control, the better the control effect.

In Figure 9, during the occurrence and outbreak stage of public opinion, the number of people interested in public opinion is on the rise. Therefore, if people want to limit the spread of certain rumors, they must minimize the duration of these two phases. The measures include 3 points. 1. The traditional media should quickly follow up the investigation and expose the cause of the incident as soon as possible. 2. Officials should come forward to clarify the facts as soon as public opinion erupts and reduce the spread of rumors. 3. The dissemination nodes and forwarding volume of positive public opinion should be further increased so that the whole time can be displayed in front of netizens as soon as possible to reduce the spread of rumors.

## 4. Conclusions

With the continuous development of network social media, public opinion guidance faces a more complex and changeable environment, which needs the joint management of the public, public opinion leaders, mainstream media, and the government. Here, the SIR model is adopted to study the communication control of network public opinion. By quantifying the communication problem, the communication law of the model is understood in detail, which lays a foundation for the management of network public opinion. Moreover, feasible control strategies are put forward to facilitate network public opinion communication control. In addition, a network public opinion risk management system is proposed using network public opinion risk management technology and blockchain technology to investigate network public opinion risk identification, risk association tree, and smart contract. However, there are still some deficiencies in this study. Due to the limitations of research conditions and research ability, to facilitate the calculation of the model, the change in group size is not considered, which should be taken into account in subsequent research. In addition, the treatment of latent individuals is relatively simple. They are identified as mutants with a certain probability, without considering the diversification transformation caused by individual differences. The shortcomings of this work will be studied in the future.

## Figures and Tables

**Figure 1:** Characteristics of network public opinion and the evolution mechanism of network public opinion ((a) characteristics of network public opinion; (b) evolution mechanism of network public opinion).

**Figure 2:** Schematic diagram of network public opinion dissemination.

**Figure 3:** Conceptual framework of the network public opinion risk management system.

**Figure 4:** Network public opinion early warning system.

**Figure 5:** Public opinion risk association tree.

**Figure 6:** Results of social network public opinion diffusion operation. (a) Online cultural publicity rate; (b) influence of opinion leaders; (c) sensitivity to public opinion events; and n is the control coefficient.

**Figure 7:** Track of network public opinion propagation without control. (a) The susceptible people; (b) lurker infection; and (c) infection.

**Figure 8:** Network public opinion propagation track. (Cost weight coefficient in objective function *α* is 2, UCL *u*_max_ = 0.1.) (a) The susceptible people; (b) lurker infection; and (c) infection.

**Figure 9:** Network public opinion propagation track. (Cost weight coefficient in objective function *α* is 2, UCL *u*_max_ = 0.3.) (a) The susceptible people; (b) lurker infection; and (c) infection.

## Data Availability

The data used to support the findings of this study are included within the article.
